# Application Value of Management Model Based on “Zero Tolerance” Concept in Pressure Ulcer Management

This article has been retracted.

**DOI:** 10.1155/2022/6792584

**Published:** 2022-10-10

**Authors:** Yufei Liu, Changming Zhou, Nan Li, Xiaoxue Gong

**Affiliations:** ^1^Department of Emergency Intensive Care, The Second Hospital of Dalian Medical University, Dalian 116023, Liaoning, China; ^2^Department of Invasive Technology, The Second Hospital of Dalian Medical University, Dalian 116023, Liaoning, China

## Abstract

**Background:**

Pressure injuries are the most prevalent health problem worldwide. Improving the quality of hospital pressure injury management is an important indicator to improve the quality of hospital management.

**Objective:**

To explore the application value of the management model centered on the concept of “zero tolerance” in the management of pressure ulcers (PU).

**Methods:**

The effects of conventional management mode and management mode centered on the concept of “zero tolerance” on PU patients and nursing staff were retrospectively analyzed. The patients were evaluated by the general comfort questionnaire (GCQ), Generic Quality of Life Inventory 74 (GQOL-74), and pressure ulcer healing scale (PUSH). At the same time, the satisfaction of PU patients and nursing staff with different management modes was investigated.

**Results:**

When comparing the conditions of patients under different management modes, it was found that the “zero tolerance” management mode can improve the comfort and quality of life of patients during hospitalization. Compared with the conventional management mode, the “zero tolerance” management mode can significantly improve the degree of pressure ulcer healing in patients. In addition, the “zero tolerance” management model can not only improve the satisfaction of patients with management but also improve the satisfaction of nursing staff with management.

**Conclusion:**

Standardized management of PU patients with the concept of “zero tolerance” as the core can improve the health status and quality of life of patients, promote wound healing, and improve the satisfaction of patients and nurses with the management plan.

## 1. Introduction

Pressure ulcers (PUs), formerly known as pressure injury (PI), refer to localized damage to the skin or subcutaneous tissue caused by pressure combined with shearing force, usually occurring at the bony prominence [1–3]. PU is the most prevalent health problem worldwide and has been designated by several countries as one of the most important sentinel events in healthcare [4, 5]. The place where PU occurs is uncertain, and it can occur outside the hospital, after admission, or even during transport. Pressure injury has the characteristics of long cycle, high cost and serious consequences, and has caused adverse effects on patients, patient families, medical institutions, and society [6–8].

From the patient's perspective, PU can cause pain, both during dressing changes and at rest. It has been reported that more than 65 percent of patients with PU report that pain from pressure injury has had a severe adverse effect on their daily living, mobility, and sleep [9, 10]. In addition, about 30% of PU patients have experienced emotional problems such as self-isolation, social fear, and low self-esteem due to the disordered image of patients caused by PU [11, 12]. If the pressure injury is not taken timely and effective care measures, it will lead to a series of complications such as bacterial infection and osteomyelitis. This is not only detrimental to wound healing but also can cause sepsis or cancer due to secondary infection, which is life-threatening [13, 14]. From the perspective of the patient's family, most pressure injury patients lack self-care ability due to limited activities, and their wound healing cycle is long. In addition, a patient's pressure injury imposes a significant financial cost on the family, including moist healing dressings, stress reduction equipment, new technologies and therapies, and nutritional supplements. From the perspective of medical institutions and society, stress injuries not only increase the workload of nurses in medical institutions by nearly 50% but also bring enormous economic pressure to the health care system and society [15]. In view of this, the prevention of pressure injury has become the focus of clinical nursing work, and the management of PU has also become an important part of contemporary hospital management.

“Zero tolerance” means zero and no tolerance for errors or potential pitfalls. It is the essence of the “Broken Window Theory” proposed by American political scientist James Wilson and criminologist George Kaelin [16]. The “zero tolerance” management concept tells us that small incidents and small details that are easily overlooked may lead to some major problems and should be prevented at the beginning of the incident to avoid bad hinting effects or blind obedience [17]. When implementing “zero tolerance,” it is necessary to effectively unify “prevention” and “governance,” nip the signs of violations in the bud, and improve the quality of management. The “zero tolerance” management concept is often used in the management of large industrial enterprises and is less used in medicine. This study aims to explore the application effect of the concept of “zero tolerance” in pressure injury management and provides guidance for improving the quality of pressure injury management in hospitals.

## 2. Materials and Methods

### 2.1. General Information

The clinical data of patients hospitalized in our hospital from January 2018 to December 2021 were retrospectively analyzed. Among them, our hospital implemented the conventional management model from January 2018 to December 2019 and implemented the “zero tolerance” management model from January 2020 to December 2021. The inclusion criteria of the PU patients are as follows: (1) should meet the relevant diagnostic criteria for pressure injury; (2) be awake and have the ability to communicate and communicate independently; and (3) should have complete clinical data required for this study. Exclusion criteria are as follows: (1) with contraindications to turning over; (2) transferred to hospital during treatment; (3) with mental illness; and (4) with severe skin disease or extensive skin ulceration.

Among the final included research subjects, 175 cases received the conventional management mode (referred to as the conventional group), and 180 cases received the “zero tolerance” management mode (referred to as the innovative group). The general data of patients under different management modes are shown in Table 1. After statistical analysis, it was found that the data of the two groups were balanced and comparable. In addition, the basic situation of nursing staff under different management modes was counted, including 68 nursing staff in the period of implementing the conventional management mode and 72 nursing staff in the period of implementing the “zero tolerance” management mode. After comparative analysis, it was found that the baseline data of nurses under different management modes were also balanced and comparable, as shown in Table 2. It is worth noting that the sample size of the conventional group and the innovative group in this study is slightly different because this study is a retrospective analysis and collected actual patients and nursing staff in our hospital. Although the sample sizes of the two groups were slightly different, the differences were small, and the baseline data of the two groups were balanced and comparable (Tables 1 and 2). Therefore, small differences in sample size do not affect the experimental results.

### 2.2. Management Plan

Routine management mode is as follows: (1) nursing staff inform patients and their families about pressure injury; (2) patients follow doctor's orders to cooperate with physicians in pressure injury treatment and care; (3) pay attention to changes in patients' physical signs and wound healing; (4) keep the ward environment clean and the beds clean and tidy, and regularly assist patients to turn over and change their clothes; (5) instruct patients to eat scientifically, and inform their family members of daily nursing precautions.

Management model based on the concept of “zero tolerance.” The specific contents of the “zero tolerance” management model are as follows: (1) to train the nurses in the department on the “zero tolerance” management concept and to evaluate the participants. Promote the training staff to pay attention to the management of stress injury and enhance the initiative of management. (2) Through regular inspections and special personnel responsibility system, we can timely find out the bad phenomena in the management. Medical staff should formulate measures and intervene in time for potential risk factors, and never let go of any adverse phenomena that may cause management problems. Hospital managers should also pay enough attention to accidental adverse phenomena and minor faults to ensure timely elimination of potential hidden dangers. (3) The problems in nursing work should be recorded and analyzed in time, and relevant meetings should be organized to discuss the reasons for the problems. Based on the results of the analysis, we will improve the management of pressure injury, scientifically optimize the management process, and constantly update the management standards. (4) For possible serious situations, an emergency response plan should be formulated in advance, and the emergency response plan should be exercised in advance to ensure the nursing staff's ability to deal with emergencies. (5) Strengthen the effective management of pressure injury through continuous improvement of management measures, improve the management awareness of relevant nursing staff, and ensure the quality of nursing.

### 2.3. Observation Indicators

(1) The comfort state of the patients was assessed by the general comfort questionnaire [18] (GCQ). The GCQ includes 4 dimensions of physiology, psychology, spirit, social culture, and environment, with a total of 28 items (10 positive rating items and 18 negative rating items). All items were scored using a 4-level scoring method, with a total score ranging from 4 to 112, with higher scores indicating higher comfort. (2) Generic Quality of Life Inventory 74 [19] (GQOL-74) was used to assess the quality of life of patients. GQOL-74 has a total of 74 items, and it evaluates the health-related quality of life of the respondents from four dimensions: physical function, psychological function, social function, and material life status. Each functional dimension score and total score of GQOL-74 were converted into a range of 0 to 100, with higher scores indicating better quality of life. (3) The pressure ulcer healing score scale [20] (PUSH) was used to evaluate and compare the management effect of the two groups of patients. The PUSH scale can comprehensively evaluate the pressure injury of PU patients from the area of pressure ulcer, the amount of exudate, and the type of wound tissue. The total score of PUSH scale ranges from 0 to 17, with lower scores indicating better wound healing in PU patients. (4) Self-made satisfaction scale was used to evaluate the satisfaction of patients and nurses with the management plan. The satisfaction level is divided into four levels: very satisfied, relatively satisfied, basically satisfied, and not very satisfied.

### 2.4. Statistical Analysis

The data of this study were analyzed using SPSS 25 and GraphPad 8.3 statistical software. Quantitative data conforming to a normal distribution were expressed as ($\bar{x}\pm s$), and differences between groups were tested by *t*-test. Categorical data were represented by *n* (%), *χ*^2^ test was used for comparison between two groups, and rank sum test was used for rank data. The comparison of all data indicated that the difference was significant at *P* < 0.05.

## 3. Results

### 3.1. Comparison of GCQ Scores

When comparing the GCQ scores of patients under different management modes, it was found that after the intervention, the GCQ scores of patients who received different management modes were improved compared with those at the time of admission. Also, the GCQ scores of patients who received “zero tolerance” management were greatly higher than those of patients who received the conventional management (*P* < 0.05). The detailed data are shown in Table 3, and these results suggest that a management model based on the concept of “zero tolerance” can help improve the comfort of PU patients during hospitalization.

### 3.2. Comparison of GQOL-74 Scores

When comparing the GQOL-74 scores of patients under different management modes, it was found that after intervention, the GQOL-74 scores of patients who received different management modes were improved compared with those at admission. Also, the GQOL-74 scores of patients who received the “zero tolerance” management were greatly higher than those of patients who received routine management (*P* < 0.05). Detailed data are shown in Table 4, and these results suggest that a management model based on the concept of “zero tolerance” can help improve the quality of life of PU patients.

### 3.3. Comparing the Management Effects of Different Management Modes on Patients

The management effect of different management modes on PU patients was evaluated by the pressure ulcer healing score scale. As shown in Table 5 and Figure 1, after one week of intervention, the PUSH scores of patients who received the “zero tolerance” concept management were greatly lower than those who received conventional management (*P* < 0.05). After 2 weeks of intervention, the PUSH scores of the two groups of patients continued to decline, and the change trend was the same as that after 1 week of intervention.

### 3.4. Patient and Caregiver Satisfaction with the Management Program

Investigate the degree of satisfaction of patients with the management plan under different management modes. After comparison, the satisfaction of the two groups of patients with the management plan under different management modes was evaluated (*Z* = −2.501, *P* = 0.012). Among them, “zero tolerance” management patients had greatly higher rates of very high satisfaction than those who received conventional management, as shown in Table 6.

Investigate the satisfaction degree of nursing staff to the management scheme under different management modes. After comparison, the satisfaction of the two groups of nursing staff with the management scheme under different management modes was evaluated (*Z* = −1.987, *P*=0.047). Nurses under the “zero tolerance” management mode were greatly more satisfied with the management scheme than those under the conventional management mode, see Table 7.

## 4. Discussion

The multiple hazards brought about by pressure injuries alert clinical medical workers to prevent the occurrence of pressure injuries. However, in clinical practice, most patients bring pressure injuries outside the hospital [21]. Patients with prehospital pressure injuries were more likely to have their condition worsened due to lower levels of self-management. Therefore, effective management of patients with existing pressure injuries on admission has become the focus of clinicians. In the management of PU patients, there are many factors that lead to the deterioration of the patient's condition or poor treatment effect, and it is necessary to explore and optimize the entire management process [22]. In the process of improper management, there is not only a lack of staff's sense of responsibility and management awareness but also a lack of patients' own awareness of the disease. These are the hidden dangers of effective management of PU patients and also the reasons for the poor treatment effect of patients. In the management of PU patients, a little management negligence may bring about huge problems in management. If the management process optimization and details are not strengthened, it is easy to cause the patient's condition to deteriorate and cause unnecessary doctor-patient disputes.

In this study, the “zero tolerance” management concept was introduced into the management of PU patients, and the management process of “nursing staff training, hidden danger inspection, cause analysis, development of plans, and improvement plans” was strictly implemented. Adhering to the concept of “zero tolerance” in the implementation process, on the one hand, it can improve the self-discipline of nursing staff and avoid adverse events caused by the negligence of nursing staff. On the other hand, it can also enhance the responsibility of the nursing staff and improve the quality of care for PU patients. This study found that under the management model based on the “zero tolerance” concept, the health status, quality of life, and wound healing of PU patients were significantly improved. As a new management model, the management model based on the concept of “zero tolerance” is an extension and optimization of traditional management. It can find out the problems in the nursing process in time, and through discussion and analysis, so as to obtain the solution to the problem. In addition, the management model based on the concept of “zero tolerance” emphasizes continuous improvement of nursing management. That is, from problem finding to problem solving, a periodic method of finding and solving problems is formed, thereby improving the quality of care.

The results of this study showed that after the implementation of the management model based on the “zero tolerance” concept, the satisfaction of both patients and nurses was significantly improved. This study believes that nursing satisfaction is an important content in the evaluation of nursing quality and hospital management quality. Scholars such as Alıcı [23] also indicated in their studies that individualized nursing satisfaction affects the quality of life of patients with the same results. In addition, scholars such as Gniadek [24] also believe that satisfaction with nursing can check the quality of medical services. It is worth noting that after the implementation of the management model based on the concept of “zero tolerance,” not only the satisfaction of patients with management has been significantly improved but also the satisfaction of nursing staff with the management plan. Nursing staff has high satisfaction with the management plan, which not only helps to improve the quality of nursing care for patients but also helps to improve the service quality of the whole hospital.

## 5. Conclusion

In this study, the application of “zero tolerance” management concept in the management of PU patients can significantly improve the health status of PU patients and promote the healing of patients' wounds. In addition, management programs based on the concept of “zero tolerance” can also improve the satisfaction of patients and caregivers with management work. Therefore, we believe that standardized management of patients with pressure injury based on the concept of “zero tolerance” can improve the health status and quality of life of patients, promote wound healing, and improve the satisfaction of patients and nursing staff with the management program.

## Figures and Tables

**Figure 1:** Comparison of management effects.

**Table 1:** Comparison of general data of patients under different management modes.

Factor	Conventional (*n* = 175)	Innovative (*n* = 180)	*χ* ^2^/*t*	*P*
Gender			0.168	0.682
Male	101 (57.71)	100 (55.56)		
Female	74 (42.29)	80 (44.44)		
Age (years)	64.28 ± 5.16	65.31 ± 5.49	1.820	0.069
BMI (kg/m^2^)	25.26 ± 1.12	25.09 ± 1.08	1.456	0.146
Staging of pressure injuries			1.725	0.631
I	58 (33.14)	66 (36.67)		
II	41 (23.43)	35 (19.44)		
III	39 (22.29)	46 (25.56)		
IV	37 (21.14)	33 (18.33)		

**Table 2:** Comparison of general data of nursing staff under different management modes.

Factor	Conventional (*n* = 68)	Innovative (*n* = 72)	*χ* ^2^/*t*	*P*
Gender			0.501	0.419
Male	7 (10.29)	5 (6.94)		
Female	61 (34.86)	67 (93.06)		
Age (years)	28.16 ± 3.19	27.62 ± 3.47	0.957	0.340
Education level			0.654	0.419
College	36 (52.94)	43 (59.72)		
Undergraduate and above	32 (18.29)	29 (40.28)		
Job title			0.914	0.339
Primary	45 (66.18)	42 (58.33)		
Intermediate and above	23 (13.14)	30 (41.67)		

**Table 3:** Comparison of GCQ scores.

Group	*n*	Before intervention	After intervention	*t*	*P*
Conventional	175	65.15 ± 9.16	76.92 ± 8.33	12.580	<0.001
Innovative	180	64.33 ± 10.09	85.17 ± 7.79	21.930	<0.001
*t*		0.801	9.641		
*P*		0.424	<0.001		

**Table 4:** Comparison of GQOL-74 scores.

Group	*n*	Before intervention	After intervention	*t*	*P*
Conventional	175	57.61 ± 5.17	66.90 ± 6.31	15.070	<0.001
Innovative	180	56.92 ± 5.63	72.65 ± 6.99	23.510	<0.001
*t*		1.202	8.128		
*P*		0.230	<0.001		

**Table 5:** Comparison of management effects.

Group	*n*	Before intervention	After 1 week of intervention	After 2 weeks of intervention
Conventional	175	11.67 ± 2.48	10.16 ± 2.16	9.42 ± 1.86
Innovative	180	11.32 ± 2.51	9.58 ± 2.08	8.13 ± 1.65
*t*		1.321	2.577	6.917
*P*		0.187	0.010	<0.001

**Table 6:** Comparison of patient satisfaction with different management programs.

Group	*n*	Very satisfied	Relatively satisfied	Basically satisfied	Not so satisfied
Conventional	175	81 (46.29)	53 (30.29)	33 (18.86)	8 (4.57)
Innovative	180	101 (56.11)	59 (32.78)	15 (8.33)	5 (2.78)
*Z*		−2.501			
*P*		0.012			

**Table 7:** Comparison of nursing staff's satisfaction with different management programs.

Group	*n*	Very satisfied	Relatively satisfied	Basically satisfied	Not so satisfied
Conventional	68	33 (48.53)	14 (20.59)	12 (17.65)	9 (13.24)
Innovative	72	45 (62.50)	16 (22.22)	6 (8.33)	5 (6.94)
*Z*		−1.987			
*P*		0.047			

## Data Availability

The data used to support the findings of this study are available from the corresponding author upon request.
